# Atrial Fibrillation Detection with Low Signal-to-Noise Ratio Data Using Artificial Features and Abstract Features

**DOI:** 10.1155/2023/3269144

**Published:** 2023-01-21

**Authors:** Zhe Bao, Dong Li, Shoufen Jiang, Liting Zhang, Yatao Zhang

**Affiliations:** ^1^School of Mechanical, Electrical and Information Engineering, Shandong University, Weihai 264209, China; ^2^School of Business, Shandong University, Weihai 264209, China; ^3^Department of Electrocardiographic, Shandong Provincial Hospital Affiliated to Shandong University, Jinan 250021, China

## Abstract

Detecting atrial fibrillation (AF) of short single-lead electrocardiogram (ECG) with low signal-to-noise ratio (SNR) is a key of the wearable heart monitoring system. This study proposed an AF detection method based on feature fusion to identify AF rhythm (A) from other three categories of ECG recordings, that is, normal rhythm (N), other rhythm (O), and noisy (∼) ECG recordings. So, the four categories, that is, N, A, O, and ∼ were identified from the database provided by PhysioNet/CinC Challenge 2017. The proposed method first unified the 9 to 60 seconds unbalanced ECG recordings into 30 s segments by copying, cutting, and symmetry. Then, 24 artificial features including waveform features, interval features, frequency-domain features, and nonlinear feature were extracted relying on prior knowledge. Meanwhile, a 13-layer one-dimensional convolutional neural network (1-D CNN) was constructed to yield 38 abstract features. Finally, 24 artificial features and 38 abstract features were fused to yield the feature matrix. Random forest was employed to classify the ECG recordings. In this study, the mean accuracy (Acc) of the four categories reached 0.857. The *F*_1_ of N, A, and O reached 0.837. The results exhibited the proposed method had relatively satisfactory performance for identifying AF from short single-lead ECG recordings with low SNR.

## 1. Introduction

Atrial fibrillation (AF) is a disordered and rapid atrial electrical activity characterized by supraventricular tachyarrhythmia. Its incidence increases with age, and millions of people are affected by AF every year [1]. In practice, real-time monitoring of cardiovascular disease is essential for early warning of AF. At present, wearable electrocardiogram (ECG) monitoring is the mainstream real-time monitoring system [2], which can help patients get rid of discomfort and time and place restrictions in the process of long-term health monitoring. However, the ECG recordings collected by wearable devices or mobile phones are easily contaminated by the complex external environment so that their signal-to-noise ratio (SNR) is low. Actually, many recordings with low SNR cannot be used for diagnosis because of their poor quality. Thus, the ECG recordings with low SNR also should be identified to avoid wasting clinical resources.

Traditional machine learning algorithms based on statistics were extensively used for data analysis [3–6]. Most of the current studies on AF automatic analysis do not focus on recognizing the noisy ECG recordings with low SNR. Krasteva et al. [3] used the limited feature set and combined with the optimized artificial neural network to conduct four-classification research on the CinC 2017 database. Goodfellow et al. [4] extracted three types of features, that is, template features, RRI features, and full waveform features using step-by-step machine and classified the CinC 2017 database into four categories. In general, previous studies can be divided into machine learning methods based on prior knowledge extracting artificial features and deep learning methods based on neural networks. Bin et al. [5] extracted 30 features including AF features, morphological features, and RR interval features from ECG recordings and trained a decision tree model using AdaBoost.M2 algorithm to realize AF detection. Datta et al. [6] extracted several categories of AF features, that is, morphological features, HRV, frequency domain, and statistical features from PhysioNet/CinC Challenge 2017 database. They first transformed a four-classification problem into two binary classification problems because the performance of binary classifier is better than that of single multi-class classifier and then used a binary classifier to classify the two binary classification problems. Finally, the ECG recordings were divided into four categories, that is, normal, AF, other, and noisy ECG recordings. Pham et al. [7] first generated third-order cumulant images from four categories of ECG recordings and extracted 18 features including entropy features and other texture-based features. They used multiple classifiers to classify the recordings into four categories, that is, *N*_sr_, *V*_fib_, *A*_fl_, and *A*_fib_. The results exhibited random forest achieved the best performance than other algorithms, that is, KNN, J48 DT, PART rules, MLP, logistic regression, and Gaussian naive Bayes. Parsi et al. [8] extracted seven new features using the Poincare representation of the R-R interval series and fused the new features with classical features to predict the paroxysmal AF. Yue et al. [9] used frequency slice wavelet transform (FSWT) to analyze the ECG segments and converted the obtained two-dimensional (2-D) time-frequency matrix into a one-dimensional (1-D) feature vector. Finally, five machine learning methods were compared to classify AF, among which the Gaussian-kernel support vector machine has the best classification performance. The classical methods need a lot of artificial features that rely on the researchers' experience. However, more artificial features are not always better because some are redundant and may even descend classification accuracy.

Another method based on convolutional neural network (CNN) is widely used in physiological signal analysis [10, 11]. CNN can acquire implicit and abstract features within the ECG recordings by the convolutions of various structures without human intervention. Kachuee et al. [12] proposed a deep CNN model for heartbeat classification, which can accurately classify five different arrhythmias with the AAMI EC57 standard. Andersen et al. [13] proposed an end-to-end method combining recurrent neural network (RNN) and CNN to extract depth features from RR interval and divide the ECG recordings into AF and normal categories. Wang [14] designed an 11-layer network architecture based on CNN and Elman neural network to realize AF detection. By comparing several advanced classification methods, the combination of the two deep neural networks was confirmed to be feasible. Fan et al. [15] designed a multiscale fusion CNN structure to divide the ECG recordings into AF and normal categories. They used filters of different sizes to obtain features of different scales from 1-D ECG recordings and classified the recordings after feature fusion. Zhang et al. [16] proposed a global hybrid multiscale CNN which can fully extract features to realize the categories of AF and normal recordings. Acharya et al. [17] designed a 9-layer CNN model to automatically identify five heartbeat categories in ECG recordings, and they also tested the model in an original recording group and a noise attenuation recording group.

Actually, with the adoption of wearable devices and mobile phones, the ECG recordings collected using the devices are easy to be contaminated by noise so that the recordings cannot be used for clinical purpose because of their poor quality. So, the noisy ECG recordings should be recognized before diagnosing. Thus, it is necessary to distinguish the acceptable ECG recordings and the noisy ECG recordings from a large lot of ECG recordings with low SNR. In previous studies, entropy helped identify the inherent nonlinear property within the ECG recordings and randomness [18]. Zhang et al. [19] calculated a multiscale entropy of the ECG recordings for signal quality assessment and further studied the sensitivity of multiscale entropy on the ECG recordings with noise. Pham et al. [7] extracted a large number of entropy features to train classifiers. Fu et al. [20] extracted different entropy features, that is, approximate entropy, sample entropy, and fuzzy entropy to feed into machine learning, that is., support vector machine (SVM), least-squares SVM (LS-SVM), and long short-term memory (LSTM) for assessing the quality of the ECG recordings. Zhang et al. [21] proposed a permutation ratio entropy (PRE) based on permutation entropy to identify random components and inherent irregularities within time series. The studies exhibited a satisfying performance of entropy methods for identifying random components and inherent irregularities within the recordings. Thus, this study used the entropy feature, namely, PRE, to identify the noisy ECG recordings and other ECG recordings.

So, a novel method was proposed in this study, which used feature fusion including artificial features and abstract features to extract comprehensive information within the ECG recordings, and the entropy feature was also employed to improve classification performance of the method for noisy ECG recordings. In this study, Section 2 introduces materials and methods, including data preparation, feature extraction, and network architecture.  Section 3 shows the results of this research.  Section 4 discusses the effectiveness of this proposed method.  Section 5 summarizes this work.

## 2. Materials and Methods

### 2.1. Database

The publicly available database provided by PhysioNet/CinC Challenge 2017 (CinC 2017) was used in this study, and it contains four categories of ECG recordings, that is, normal rhythm (N), AF rhythm (A), other rhythm (O), and noisy (∼) ECG recordings. This database consisted of 8528 single-lead ECG recordings ranging in length from 9 s to over 60 s and the ECG recordings sampled at 300 Hz [22]. All recordings were identified by the clinical experts and technicians. Among them, 5076 ECG recordings were marked as N, 758 ECG recordings were marked as A, 2415 ECG recordings were marked as O, and 279 ECG recordings were marked as ∼. These ECG waveforms are shown in Figure 1.

This study used a data-balanced method based on the imbalance of ECG recordings length, and the method effectively retained the critical information of the ECG recordings [23]. A QRS complex location algorithm was used to locate the complex position and made the recording length consistent by copying, cutting, and symmetry. In this study, all recordings were segmented or filled to 30 s. Among them, the ECG recordings with lengths greater than 30 s were randomly segmented. The recordings with lengths less than 30 s were first located to the QRS complex using the Pan–Tompkins algorithm, then the initial downward deflection in the QRS complex was determined as the starting point of the complex, and finally the recording from the starting point of the first QRS complex to the starting point of the last QRS complex was intercepted and copied until the recording length was 30 s. After unifying the length of all segments, nearly 80% of the segments were used as training set and the remaining 20% as the test set. The performance of the proposed classification method was evaluated using the remaining segments.  Table 1 shows the details of the CinC 2017 database used in this study.

### 2.2. Outline of the Proposed Method

In this study, the ECG recordings were first unified to the length of 30 s. Then, 62 features were calculated, including 24 artificial features, that is, 8 waveform features, 11 interval features, 4 frequency-domain features, and 1 nonlinear feature and 38 abstract features extracted by a 13-layer 1-D CNN. The abstract and artificial features constituted a feature vector for yielding the fused feature matrix. Finally, a random forest [24] containing 300 decision trees was employed to classify the AF segments.  Figure 2 shows the flowchart of the proposed method.

### 2.3. Artificial Features

In the field of machine learning, the use of artificial features is essential. Based on a large number of previous studies, this study used four types of features, that is, waveform features, interval features, frequency-domain features, and nonlinear feature without discarding prior knowledge, and 24 specific features were calculated [4–8].  Table 2 shows the artificial features used in this study.

#### 2.3.1. Waveform Features

In most cases, the number and amplitude of *R* waves within the four categories of ECG segments are significantly different, so the features based on the number and amplitude of *R* waves were first calculated. The Pan–Tompkins algorithm [25] was used to locate the *R* waves of all ECG segments. Then, the number of *R* waves and amplitude of all *R* waves were obtained by the location of *R* waves. Finally, the number of *R* waves was taken as one of the features, and the basic amplitude features, that is, maximum, minimum, mean, and median of *R* wave, in each segment were calculated according to the amplitude of all *R* waves. Suppose that there are *N* pieces of *R* waves in the time series. The *r* represents the amplitude of *R* wave. Therefore, the amplitude of all *R* waves is defined as [*r*_1_, *r*_2_, *r*_3_……*r*_*N*_], so the maximum value of the amplitude is [*r*_1_, *r*_2_, *r*_3_……*r*_*N*_]_max_, the minimum value is [*r*_1_, *r*_2_, *r*_3_……*r*_*N*_]_min_, and the mean value is [*r*_1_, *r*_2_, *r*_3_……*r*_*N*_]_median_.

In the analysis of time series, many time series exhibit irregular distribution. Still, the distribution of the mean of the series shows a certain regularity, which requires that we must have an indicator to measure the relationship between each point in the series and the mean. So, the standard deviation was used to distinguish the pseudo law of distribution in this study. Another waveform feature, namely, the feature based on standard deviation, was also calculated in this study. Suppose the time series with *N* points is defined as [*X*_1_, *X*_2_, *X*_3_……*X*_*N*_], and their mean value is *‾X*. The standard deviation (*S*) is calculated as the following:

(1) $$\begin{array}{c} S=\sqrt{\frac{\overset{N}{\underset{i=1}{\sum }}{\left(X_{i}-\bar{X}\right)}^{2}}{N}}\text{,} \end{array}$$

where *i* takes a non-negative integer and starts from 1 until *N.* According to the definition of *S*, the amplitude standard deviation is also calculated as one of the waveform features.

Based on the standard deviation, the skewness (SK) and kurtosis (KU) of the segments were calculated. SK represents the characteristic number of the asymmetry degree of the probability density distribution curve relative to the average value, and KU represents the characteristic number of the peak height of the probability density distribution curve at the average value. SK is calculated as the following:

(2) $$\begin{array}{c} \begin{array}{c} SK=\frac{\overset{N}{\underset{i=1}{\sum }}{\left(X_{i}-\bar{X}\right)}^{3}}{\left(N-1\right)S^{3}} \end{array}\text{.} \end{array}$$

KU is calculated as the following:

(3) $$\begin{array}{c} KU=\frac{\overset{N}{\underset{i=1}{\sum }}{\left(X_{i}-\bar{X}\right)}^{4}}{\left(N-1\right)S^{4}}-3\text{.} \end{array}$$

To sum up, 8 waveform features were extracted from the ECG segments.

#### 2.3.2. Interval Features

RR interval refers to the duration between two adjacent *R* waves in ECG, and it can reflect the duration of one heart contraction. These features of RR interval can reflect whether a person's heart rate is normal, so heart rate can be calculated by the RR interval [26]. The heart rate of patients with AF or other abnormal hearts may be irregular, and the RR interval may be too large, too small, or unstable. Therefore, the relevant features of RR interval, that is, maximum, minimum, mean, median, and standard deviation of RR interval were calculated, and the heart rate was also obtained from the RR interval as a feature.

Heart rate (HR) is calculated as the following:

(4) $$\begin{array}{c} HR=\frac{60}{\bar{R}}\text{.} \end{array}$$

PR interval refers to the time interval from the starting point of the *P* wave to the starting point of the QRS complex on ECG. Some studies have used and proved the effectiveness of PR interval for ECG classification [3, 27, 28]. To get the PR interval, the *P* wave of the ECG recording should be located. *P* wave is easy to detect in regular ECG recordings, but it is difficult to detect in noise environment because the change is not obvious. Therefore, we used the *P*-wave detection method based on wavelet transform proposed by Li et al [29]. The PR interval was then calculated. Too long, too short, or variable PR interval represents different conditions of patients. Considering that there may be different situations for separating other classes in this database to locate these situations to the greatest extent, the relevant features of PR interval, that is, maximum, minimum, mean, median, and standard deviation of PR interval were extracted in this study. The calculation methods of relevant features of PR interval are the same as that of RR interval.

Finally, 6 features of RR interval and 5 features of PR interval were extracted from the ECG segments.

#### 2.3.3. Frequency-Domain Features

In most of machine learning methods, frequency-domain features are usually used to reflect frequency and energy information within the ECG recordings. In medical diagnosis or other application scenarios, it can be used as a part of the feature vector together with time-domain features and other features to enrich the types of feature quantities and improve the diagnostic accuracy [30]. In this study, Fourier transform, a simple spectrum analysis method, was selected to obtain the spectrum of the ECG segments and the four frequency-domain features, that is, frequency center of gravity, mean-square frequency, root mean square frequency, and frequency variance were received and applied to this study.

Assuming the frequency function is *S* (*f*), and *S* represents the spectrum and *f* represents the frequency of the segment. The frequency center of gravity (FC) is calculated as follows:

(5) $$\begin{array}{c} FC=\frac{\int_{0}^{\infty }fS\left(f\right)df}{\int_{0}^{\infty }S\left(f\right)df}\text{.} \end{array}$$

The mean-square frequency (MSF) is calculated as follows:

(6) $$\begin{array}{c} MSF=\frac{\int_{0}^{\infty }f^{2}S\left(f\right)df}{\int_{0}^{\infty }S\left(f\right)df}\text{.} \end{array}$$

The root mean square frequency (RMSF) is calculated as follows:

(7) $$\begin{array}{c} RMSF=\sqrt{MSF}\text{.} \end{array}$$

The frequency variance (FV) is calculated as follows:

(8) $$\begin{array}{c} FV=\frac{\int_{0}^{\infty }{\left(f-FC\right)}^{2}S\left(f\right)df}{\int_{0}^{\infty }S\left(f\right)df}\text{.} \end{array}$$

Finally, 4 features of frequency domain were extracted from the ECG segments.

#### 2.3.4. Nonlinear Feature

In some ECG classification studies, nonlinear features are widely used, especially various entropies are used to evaluate the complexity of signals. Many entropies, that is, Shannon entropy and permutation entropy, still cannot identify the nonlinear features in the signal. PRE was employed in the proposed method because it can identify nonlinear within ECG recordings, and the details of the PRE are in Reference [21]. This PRE can reflect the amplitude difference between two adjacent data points of a certain time series. Because it is sensitive to recording mutation and various changes, the classical permutation entropy is often used to measure the complexity of physiological recording sequence. However, the original time series cannot be measured by permutation entropy, so some details will be lost. Furthermore, permutation entropy is based on the ranking between data points, which also shows that permutation entropy ignores the differences between adjacent data points. Comparing with the classical permutation entropy, the PRE can reflect the relationship between adjacent data points by constructing the relationship matrix of adjacent elements and better reflecting the confusion degree of time series.

First, PRE constructs a new relationship matrix *B* to represent the relationship between adjacent elements and then calculates the number of new patterns *c*. Let *B* (*i*) be the *i*th row vector of matrix *B*, and *c* (*i*) be the number of the *i*th pattern. For *B* (*i*), when another vector *B* (*j*) of matrix *B* has the same mode as *B* (*i*), *c* (*i*) increases by 1, and the two have a high correlation; when each vector of matrix *B* represents a new mode, the maximum total number of mode *c* is *n* − *m* − 1. Finally, the total number of mode *c* contained in matrix *B* can be obtained.

*P *_*i*_ is the probability of pattern *c* (*i*), which is defined as the following:

(9) $$\begin{array}{c} P_{i}=\frac{c\left(i\right)}{\overset{k}{\underset{j=1}{\sum }}c\left(i\right)}\text{,} \end{array}$$

where *k* is the total number of patterns *c*, 1 ≤ *k* ≤ *n* − *m* − 1.

PRE is defined as the following:

(10) $$\begin{array}{c} PRE=-\overset{k}{\underset{j=1}{\sum }}P_{j}\ln P_{j}\text{.} \end{array}$$

### 2.4. 1-D CNN and Abstract Features

Actually, a deeper network helps to extract deeper features within ECG segments; however, the most severe problem of deeper network was to use too many parameters, which would lead to a large amount of memory and computing resources for training and interference [31]. So, a 1-D CNN was directly used to extract abstract features in this study which was constructed from six pairs of convolutional layers and a maximum pooling layer in our proposed feature extraction network.

Larger convolution kernel size had been used on the first layer of convolution layers, and the convolution kernel size rose stepwise as the number of layers increased.  Table 3 shows architecture of the 13-layer 1-D CNN and its detailed parameters. When an ECG segment was fed into the network, the segment passed through 6 pairs of convolution pooling layers. In order to obtain the abstract features, the final full connection layer changed the dimension of the output to get a 1 × 38 vector which meant 38 abstract features.

### 2.5. Fusion of Artificial and Abstract Features

Artificial features and abstract features were fused, and a feature vector of length 62 was constructed. The vector was denoted as [*R*_1_, *R*_2_, *R*_3_…*R*_24_, *S*_1_, *S*_2_, *S*_3_⋯*S*_38_]^T^. The *R*_*i*_ represents the *i*th artificial features, and *i* = 1, 2,…, 24. The *S*_*j*_ represents the *j*th abstract features, and *j* = 1, 2,…, 38. So, the feature matrix is defined as the following:

(11) $$\begin{array}{c} \left(\begin{array}{ccc} R_{1}^{1} & \cdots \cdots & R_{1}^{N}\\ \begin{array}{c} \vdots \\ R_{24}^{1}\\ S_{1}^{1}\\ \vdots \end{array} & \ddots & \begin{array}{c} \vdots \\ R_{24}^{N}\\ S_{1}^{N}\\ \vdots \end{array}\\ S_{38}^{1} & \cdots \cdots & S_{38}^{N} \end{array}\right)\text{,} \end{array}$$

where *N* represents the number of input segments.

### 2.6. Random Forest

In CinC 2017, Zabihi et al. [32] and Kropf et al. [33] used random forest to train the extracted features to obtain classification results because random forest is interpretable explain [34]. So, random forest was employed in this study. Random forest is inherited together by several decision trees. Each decision tree is a small classifier, and random forests synthesize all classification voting results to determine the final output categories.

In this study, the classification of random forest included training and testing, and the bootstrap method was used to train the random forest. In the training process, 80% of the feature vectors were used as the training set, and a group of decision trees was trained according to the tags marked in the ECG recordings. The remaining 20% was used for testing. The training process sets the maximum number of decision trees as 300, where each node randomly selected features in the generation process. Assuming that the number of the samples was *n*, the number of features in the randomly selected feature subset by the decision tree node at each segmentation was set as default, that is, the square root of the total number of features, that is, $\sqrt{n}$. The minimum number of samples required for internal node division was set as 2, the maximum depth of the decision tree was set as 40, and the training ended when the maximum depth was reached. The above parameters were set to prevent overfitting. Finally, the classification category was determined by averaging the classification voting results of all decision trees.

## 3. Results

### 3.1. Evaluation Indicators

In this study, accuracy (Acc), precision, recall, and *F*_1_ were used to evaluate performance of the proposed method.

The Acc is calculated as the following:

(12) $$\begin{array}{c} A\text{cc}=\frac{TP+TN}{TP+FN+TN+FP}\text{,} \end{array}$$

where true positive (TP) represents the number of ECG recordings in a given category that are correctly classified as the given category, false positive (FP) represents the number of ECG recordings that other categories are misclassified as the given category, true negative (TN) represents the number of ECG recordings that other categories are not classified as the given category but are classified as the correct category, and false negative (FN) represents the number of ECG recordings that other categories are not classified as the given category and are not classified as the correct category.

The precision is calculated as the following:

(13) $$\begin{array}{c} precision=\frac{TP}{TP+FP}\text{.} \end{array}$$

The recall is calculated as the following:

(14) $$\begin{array}{c} recall=\frac{TP}{TP+FN}\text{.} \end{array}$$

Like CinC 2017, the *F*_1*n*_, *F*_1*a*_, *F*_1*o*_, and *F*_1*p*_ are defined as the *F*_1_ score of the *N*, *A*, *O,* and ∼ categories, respectively, and they are calculated as the following [22]:

(15) $$\begin{array}{c} F_{1n}=\frac{2\times Nn}{\sum N+\sum n}\text{,}\\ F_{1a}=\frac{2\times Aa}{\sum A+\sum a}\text{,}\\ F_{1o}=\frac{2\times Oo}{\sum O+\sum o}\text{,}\\ F_{1p}=\frac{2\times Pp}{\sum P+\sum p}\text{.} \end{array}$$

Where *Nn, Aa, Oo, and Pp* represent the number of predicted classifications obtained by the proposed method that are consistent with the actual reference classifications of ECG recordings. ∑*N* represents the number of recordings whose reference classification is *N* and ∑*n* represents the number of recordings whose predicted classification is *N*, ∑*A* represents the number of recordings whose reference classification is *A* and ∑*a* represents the number of recordings whose predicted classification is *A*, ∑*O* represents the number of recordings whose reference classification is *O* and ∑*o* represents the number of recordings whose predicted classification is *O*, and ∑*P* represents the number of recordings whose reference classification is ∼ and ∑*p* represents the number of recordings whose predicted classification is ∼.  Table 4 clearly showed the counting rules of the above variables. The total of *F*_1_ is defined according to the rules of the CinC 2017 and it is obtained by taking the macro average of the three scores, and it is defined as the following:

(16) $$\begin{array}{c} F_{1}=\frac{F_{1n}+F_{1a}+F_{1o}}{3}\text{.} \end{array}$$

### 3.2. Results

In this study, 80% of the ECG segments were used as training set, and the rest 20% were used as test set for evaluating the proposed method. For the training set, we used 10-fold cross-validation which randomly selected 90% of the data for training and 10% for validation. The results are shown in Table 5. The corresponding recall, precision, and *F*_1_ of the *N* category achieved the highest 0.896, 0.910, and 0.913 than that of other three categories, that is, *A*, *O,* and ∼. In addition, the average of indicators of four categories, that is, recall, precision, and *F*_1_, is higher than 0.800, at 0.816, 0.813, and 0.809, respectively.

Table 6 shows a confusion matrix of the proposed method for the test set and the corresponding recall, precision, *F*_1*n*_, *F*_1*a*_, *F*_1*o*_, *F*_1*p*_, *Acc,* and *F*_1_. The *N* category yields the highest recall of 0.893, precision of 0.901, and *F*_1*n*_ of 0.901 than other categories, that is, *A*, *O,* and ∼. The ∼ category yields the lowest recall of 0.761, precision of 0.711, and *F*_1*p*_ of 0.735 among all categories. In addition, the *F*_1_ and the Acc reached 0.837 and 0.857, respectively.

Table 7 collected the results of some previous studies and compared them with the results of the proposed method. The proposed method achieved the highest Acc of 0.857, *F*_1*p*_ of 0.735 than all studies and the highest *F*_1_ of 0.837 than all studies except the *F*_1_ 0.841 of Wang et al. [35]. Actually, Wang et al. ignored the ∼ category of ECG recordings and used only three categories of ECG recordings of the CinC 2017, that is, *N*, *A,* and *O* for classification. Zihlmann et al. [39] combined LSTM and CNN to extract abstract features, and the total *F*_1_ score reached 0.820. The classification results of ∼ category in the training process were low, and the *F*_1*p*_ was only 0.645.

## 4. Discussion

### 4.1. Evaluating Effectiveness of PRE for Noisy Recording Recognition

Two feature schemes, that is, all features and all features except the PRE were compared to evaluate the effectiveness of the PRE for recognizing noisy ECG segments.  Table 8 shows the comparison results for the two feature schemes using this proposed method. The Acc of 0.857, *F*_1_ of 0.837, and *F*_1*p*_ of 0.735 for all features are higher than for all features except the PRE. The results indicate the PRE helps to classify the noisy ECG segments because the *F*_1*p*_ of 0.735 for all features is higher than the *F*_1*p*_ of 0.679 for all features without PRE. Meanwhile, a radar chart was also designed to show more clearly the differences between results of the two schemes.  Figure 3 shows a radar map of results for the two feature schemes. The *F*_1*p*_ for all features is obviously higher than that for all features except the PRE.

PRE was an improvement based on permutation entropy for identifying nonlinear chaotic character within time series instead of randomness. In PRE, a new relationship matrix *B* was constructed. This matrix was based on the relationship between adjacent elements and can closely reflect the gap between two points, especially in complex signals. The generation of the new mode *c* can avoid the repeated counting of the vector and was conducive to the complexity analysis of the whole signal. The ablation experiment showed the PRE not only played a role in noise classification but also helped the overall classification indicators.

### 4.2. Comparison of Effectiveness of Artificial, Abstract, and Fusion Features

In this study, the corresponding Accs of the three feature schemes, that is, artificial features, abstract features, and fusion features were also calculated to evaluate the effectiveness of the schemes.  Table 9 shows the corresponding Accs of artificial features, abstract features, and fusion features. The Acc of 0.820 was obtained for the scheme using only artificial features. Similarly, the Acc for only abstract features generated by the 13-layer 1-D CNN was the lowest 0.734 than that for all feature schemes.

Actually, deep learning can extract effective abstract features with the support of a large amount of data. However, the existed ECG databases are small so that deep learning algorithms cannot make full use of its power for acquiring abstract features. The artificial features were summarized on the basis of expert experience and a large number of experiments, and the features can reflect information within the ECG recordings. Therefore, abstract and artificial features were combined to make the model have the advantages of both, thus improving the classification performance of the model. After fusing artificial features and abstract features, the Acc was improved to the highest 0.857 among the Accs for all schemes. The fusion features gave full play to the advantages of the two types of features and can more comprehensively reflect the information in ECG recordings, so fusion features can improve the classification performance of such models.

## 5. Conclusions

In this study, an AF detection method that combined artificial features with abstract features was proposed, and it yielded the higher results, that is, Acc of 0.857, *F*_1_ of 0.837, and *F*_1*p*_ of 0.735 for the database provided by the CinC 2017 than the previous studies. In addition, the nonlinear feature, that is, PRE, helps to identify the noisy ECG recordings from other recordings because the PRE can identify, to some extent, nonlinear irregularities within the ECG recordings instead of randomness caused by noise. Finally, the proposed method exhibits relatively satisfied performance for the ECG recordings with low SNR.

## Figures and Tables

**Figure 1:** Examples of four categories of ECG recordings.

**Figure 2:** Flowchart of the proposed method.

**Figure 3:** Radar map of results for the two feature schemes.

**Table 1:** Details of the CinC 2017 database.

Category	Recording	Training set	Test set	Sampling frequency (Hz)	Uniform length (s)
N	5076	4101	975	300	30
A	758	619	139		
O	2415	1916	499		
∼	279	208	71		

**Table 2:** Artificial features used in this study.

Feature type	Name
Waveform features	The number of *R* wave
	Maximum amplitude of *R* wave
	Minimum amplitude of *R* wave
	Mean amplitude of *R* wave
	Median amplitude of *R* wave
	Amplitude standard deviation of *R* wave
	SK
	KU

Interval features	Maximum of RR interval
	Minimum of RR interval
	Mean of RR interval
	Median of RR interval
	Standard deviation of RR interval
	HR maximum of PR interval
	Minimum of PR interval
	Mean of PR interval
	Median of PR interval
	Standard deviation of PR interval

Frequency-domain features	FC
	MSF
	RMSF
	FV

Nonlinear feature	PRE

**Table 3:** Architecture parameters of the 1-D CNN.

No.	Layer	Kernel size	Kernel number	Stride	Output size
0	Input	—	—	—	1 × 3000
1	Convolution-1	5	4	1	4 × 2996
2	Pooling	—	—	2	4 × 1498
3	Convolution-2	5	8	1	8 × 1494
4	Pooling	—	—	2	8 × 747
5	Convolution-3	7	16	1	16 × 741
6	Pooling	—	—	2	16 × 370
7	Convolution-4	7	16	1	16 × 364
8	Pooling	—	—	2	16 × 182
9	Convolution-5	9	32	1	32 × 174
10	Pooling	—	—	2	32 × 87
11	Convolution-6	11	32	1	32 × 77
12	Pooling	—	—	2	32 × 38
13	FC	—	—	—	1 × 38

**Table 4:** Counting rules for some variables.

		Predicted classification				
Reference classification		*N*	*A*	*O*	∼	Total
	*N*	*Nn*				∑*N*
	*A*		*Aa*			∑*A*
	*O*			*Oo*		∑*O*
	∼				*Pp*	∑*P*
	Total	∑*n*	∑*a*	∑*o*	∑*p*	

**Table 5:** Results of using 10-fold cross-validation against the training set.

Label	Recall	Precision	*F*_1*n*_	*F*_1*a*_	*F*_1*o*_	*F*_1*p*_
*N*	0.896	0.910	0.913	—	—	—
*A*	0.814	0.827	—	0.806	—	—
*O*	0.808	0.788	—	—	0.795	—
∼	0.745	0.726	—	—	—	0.721
Average	0.816	0.813	0.809			

**Table 6:** Confusion matrix of 1-DCNN for test set.

True	Predicted				Recall	Precision	*F*_1*n*_	*F*_1*a*_	*F*_1*o*_	*F*_1*p*_	Acc	*F*_1_
	*N*	*A*	*O*	∼								
*N*	871	13	83	8	0.893	0.908	0.901	—	—	—	0.857	0.837
*A*	11	110	15	3	0.791	0.815	—	0.803	—	—		
*O*	72	7	409	11	0.820	0.796	—	—	0.808	—		
∼	5	2	7	54	0.761	0.711	—	—	—	0.735		—

**Table 7:** Comparison of classification results.

Author	Year	Database	Feature extraction	Task	Method	Acc	*F*_1*p*_	*F*_1_
Datta et al. [6]	2017	CinC 2017 AF DB	HRV, frequency domain, and statistical features	4-Class	Multilayer cascaded binary classifiers	—	—	0.830
Cao et al. [23]	2020	CinC 2017 AF DB	Abstract features	3-Class	2-Layer LSTM	0.844	—	0.827
Zabihi et al. [32]	2017	CinC 2017 AF DB	Time domain, frequency domain, time-frequency domain, and nonlinear features	4-Class	Random forest	—	0.504	0.830
Kropf et al. [33]	2017	CinC 2017 AF DB	Time-domain and frequency-domain features	4-Class	Random forest	—	0.648	0.830
Wang et al. [35]	2020	CinC 2017 AF DB	Abstract features	3-Class	DMSFNet	—	—	0.841
Gao et al. [36]	2021	CinC 2017 AF DB	Abstract features	3-Class	RTA-CNN	0.851	—	—
Mahajan et al. [37]	2017	CinC 2017 AF DB	Time domain, frequency domain, linear, and nonlinear features	4-Class	Random forest	—	—	0.780
Xiong et al. [38]	2017	CinC 2017 AF DB	Abstract features	4-Class	CNN	—	—	0.820
Zihlmann et al. [39]	2017	CinC 2017 AF DB	Abstract features	4-Class	CNN + LSTM	0.823	0.645	0.820
Gliner and Yanav [28]	2018	CinC 2017 AF DB	Time-frequency domain, statistical features, and morphological features	4-Class	SVM	—	—	0.800
Athif et al. [40]	2018	CinC 2017 AF DB	Statistical features and morphological features	4-Class	SVM	—	—	0.780
Chen et al. [41]	2018	CinC 2017 AF DB	Morphological features and heart rate variability features	4-Class	XGBoost	—	—	0.810
This work	2022	CinC 2017 AF DB	Time domain, interval, frequency domain, and nonlinear features and abstract features	4-Class	Fusion features + random forest	0.857	0.735	0.837

**Table 8:** Comparison results for the two feature schemes.

	Feature scheme	
	All features	All features except the PRE
Acc	0.857	0.836
*F*_1_	0.837	0.822
*F*_1*p*_	0.735	0.679

**Table 9:** Accs of three feature schemes, that is, artificial features, abstract features, and fusion features.

	Feature scheme		
	Artificial feature	Abstract feature	Fusion feature
Acc	0.820	0.734	0.857

## Data Availability

The data used to support the findings of this study are available from the corresponding author upon request.
